# Rapid Control of Government Economic Environment Management Cost Based on Balanced Score Card

This article has been retracted.

**DOI:** 10.1155/2022/8506676

**Published:** 2022-08-02

**Authors:** Yumei Wang, Zhirong Shen, Yicheng Zhou

**Affiliations:** ^1^Business School, Suzhou University of Science and Technology, Suzhou 215009, China; ^2^School of Politics and Public Administration, Soochow University, Suzhou 215123, China; ^3^Centre for Chinese Urbanization Studies, Soochow University, Suzhou 215123, China

## Abstract

EMC (economic management cost) of the government has become a hot topic of concern from all walks of life. Controlling and reducing government EMC is the requirement for building a conservation-oriented society and deepening the reform of public budget. Dynamic cost accounting calculates the cost of cost objects through the confirmation, measurement, and distribution of production costs. In this article, it is innovatively proposed to integrate BSC (balanced score card) into EMC control, and analyze the logical relationship between system objectives and functions by using the mathematical model. Based on GA (genetic algorithm) cost optimization control concept and specific control ideas, individuals who meet the evolutionary characteristics are stored in the crossover database and participate in crossover operation as parents when crossing. In order to improve the local optimization ability of the algorithm, parallel mutation operation mechanism is introduced, which can execute multiple mutation rules at the same time. The results show that the average convergence time of this algorithm is 0.186s and the variance of population fitness is 288.19. The conclusion shows that the algorithm proposed in this article can overcome the problems of slow convergence speed, low accuracy, and local convergence of GA, and effectively improve the overall performance of the algorithm.

## 1. Introduction

Cost management is currently very important due to China's economic integration and the ongoing development of the market economy. The public is becoming more and more concerned with the government's EMC (economic management cost), which is an important executor and manager of social and public activities. Anti-corruption efforts have stepped up, particularly in recent years, and the cost of government administration has gradually come under scrutiny. Future social and economic development of a nation or region is now significantly influenced by the status of the EMC government. The socialist market economic system mandates that the government increase its EMC awareness, and it is also a component of a world-compliant government operation mechanism [1]. In reality, the general lack of government awareness of EMC and its effects have put the issue of boosting government awareness of EMC on the agenda in both political and academic circles.

Government EMC departments have been actively established in all Western nations, which place great importance on government EMC research and management. According to Nuria et al., the purpose of administration research is to first understand what the government can do effectively and efficiently [2]. To analyze the strategic cost of enterprises, Nita et al. proposed using value chains [3]. The business operations of enterprises are broken down into a series of activities related to strategies through value chain analysis, greatly enhancing the operational viability of the strategic theory. The ideas of cost-leading strategy and cost differentiation strategy, among others, form the cornerstone of EMC control. BSC (balanced score card) design should be integrated with enterprise strategy, according to Pang et al. [4]. This demonstrates how the study of BSC has progressed from the discipline of performance assessment to the discipline of strategic management. Li et al. realize the strategic management function of BSC by ensuring the efficient execution of organizational strategy through the causal relationship between organizational elements. It ties employee work to government strategy and coordinates individual employee efforts to carry out government strategy [5]. EMC is a useful metric for measuring administrative effectiveness and the level of government management, and its level is directly correlated with the public's perception of the government's standing and reputation. The number of local governments in China with excessive EMC is currently growing quickly, and the public's voice in favor of reducing EMC is growing stronger.

The successful management and control of local government EMC is a great accomplishment that has both immediate and long-term advantages. No matter the time period, strict EMC regulation has always been a top priority for all tiers of government. In light of the current research on EMC, this article presents ideas and solutions for the government's quantitative EMC measurement and control practice, which is crucial for lowering EMC and enhancing administrative efficiency. Regarding government EMC, we must pay attention to both investments and results, implement private sector management, reduce government EMC in numerous ways, set up a system for assigning responsibility for government EMC, and exercise comprehensive control over government EMC.

The following aspects of this article are intended to be innovative: (1) this study investigates the internal law of EMC change in China and identifies the underlying causes of China's political issues by using analysis tools for system formation and change, transaction cost, cost-benefit, and other variables. Furthermore, new countermeasures should be proposed in order to make the analysis more accurate, objective, and useful as a reference. (2) Cost control is the main concern of businesses today, given a certain profit level. In this study, GA is used to address the best combination allocation of process costs, or best cost control. This study introduced the distinct control concept and ideas of target cost optimization control, combined them with the three major trends that are currently in place—quality control, construction period, and cost—and conducted research on the most effective control under the constraints of target cost based on GA.

## 2. Related Work

### 2.1. Government EMC Control Research

Western countries, especially European and American countries, attach great importance to the research of EMC. The American government even measures the local government's EMC on that day by the average daily wage of workers, thus playing a role in controlling and restricting EMC. Johnstone put forward the “bureaucracy” which has a far-reaching influence on administration. This system achieves the goal of maximum efficiency with a rational management organization structure, and it is especially important for EMC research [6]. Prebilic et al. revealed the current situation that the EMC of our government is too high and growing too fast, and analyzed the deep-seated reasons. After listing all kinds of reasons, they deduced the good strategies for controlling the EMC of our government one by one, and put forward the effective methods to reduce the EMC of local governments from the aspects of changing officials' ideology, streamlining the scale of personnel organizations, strengthening the supervision mechanism, and simplifying the administrative examination and approval procedures [7]. Munkratok et al. made analysis from the perspective of development, and came to an important theory: it is reasonable for administrative expenditure to keep pace with the level of economic growth. The reason is that the demand for EMC is gradually increasing with the process of economic growth [8].

Torriti et al. put forward the theory of bureaucratic budget maximization, that is, bureaucrats always pursue the maximization of total budget [9]. Furceri applied the analysis framework of cost-benefit in enterprise theory to the analysis of government management, and put forward 10 principles of transforming public sector and shaping new government with entrepreneurial spirit [10]. Kriwoluzky put forward that EMC is the social resource paid by people in the society to maintain the government's operation. In a narrow sense, it only refers to the social material resources consumed by the government, and it also refers to the fact that the government damages or abandons other value realization in order to achieve the established government value goals when exercising its due functions [11]. Benarroch et al. pointed out that improving the decision-making mechanism of local government is the basis of controlling EMC, and at the same time, strengthening the enforcement and supervision to achieve mutual checks and balances between power and supervision [12].

However, the domestic research on the definition and quantitative analysis of EMC is still inconclusive, and there is no relatively uniform standard, which still needs further integration. The feasibility and effectiveness of measures to control EMC also need more research and demonstration.

### 2.2. Research Status of BSC

BSC is now a tool for the group's strategic management and is crucial to the group's planning, execution, and management. The traditional approaches that relied primarily on financial indicators cannot satisfy the needs of businesses in the information society, and businesses must broaden their horizons to achieve their objectives. In order to establish a trustworthy performance management system based on execution and complete the system's strategic objectives, BSC breaks down the company's strategic objectives into a number of distinct and balanced performance evaluation indicators. It then assesses the realization of these indicators over time.

Lorenzon et al. explained how top managers use BSC as an important management process framework, which makes leaders have a comprehensive management tool for four key factors: planning strategy, personnel, process, and execution [13]; Huang et al., taking the case of company's implementation of BSC as the research object, clarified and analyzed the process and necessary steps of implementing organizational strategy with BSC [14]. Rajesh et al., based on the core idea of BSC, put forward a theoretical model to improve the service efficiency of bank outlets [15]. Assiri et al. comprehensively applied the relevant theories of performance appraisal and BSC to study the present situation and existing problems of employees' performance appraisal in order to stimulate employees' creativity and gain a competitive advantage for enterprises [16].

Yong et al. introduced the drawing elements, principles, and time parameters of a network diagram in detail [17], and proved that it is feasible to apply network planning technology to project schedule management for network analysis, and it is systematic, controllable, and dynamic. Debien et al. pointed out that the scheduling problem with resource constraints can only be applied to cases with less than 50 activities if the optimal solution is adopted [18]. Khanmirza et al. introduced GA (genetic algorithm) into resource optimization, and proposed a new method of effective crossover of ordered chromosomes. The mutation operator was defined by the method of searching improved offspring by combining centralized search strategy design with neighborhood technology, which solved two kinds of problems of resource optimization well [19]. Chaoui divides resources into tangible resources and intangible resources, breaking the traditional limitation of equating resources with tangible entities. An S-shaped schedule curve management method based on simulation loop network simulation technology is proposed. Under the uncertain condition, the mean and variance of each duration are statistically analyzed, and the probability distribution is obtained [20]. Ding et al. used the dynamic programming method to deal with the optimization problem of time limit and cost in the method of expressing key lines by a series of single-stage decisions [21].

## 3. Methodology

### 3.1. Government EMC Analysis

Government EMC control requires the cooperation of all government departments and cannot be done on its own. Because cost information from other departments serves as the foundation for cost control, it will be challenging to accomplish this goal. To increase the accuracy and dependability of cost control, the government should therefore improve the fundamental cost control. Public finance adheres to the market failure criterion when discussing the primary and fundamental issue of the relationship between government, finance, and the market, that is, under the circumstances of a market economy, the government and its financial public can only make the appropriate failure state for the needs of the market as their own behavior criterion. China's governments have long suffered from the drawbacks of low administrative efficiency, including large government agencies, bloated government agencies, and surplus staff, all of which significantly erode and harm administrative efficiency [2, 3].

The market's primary function in the fast-paced operation of today's market economy is basic regulation, with the government acting as a backup plan when the market falters. An essential tool for allocating money for the use of various public goods and services is the public budget. The government must decide how to prioritize allocating financial resources among competing demands. The people's congress system that governs China requires that consideration of “cost-benefit” be given priority when making administrative decisions. Cost-benefit analysis is required when using administrative resources. As a result, the EMC's control over our government complies with the reasonable demands for the reform of our economic system. The legal demand of social external demand for the supply of government institutions is a crucial criterion to assess whether the resource input demand of administrative organs is reasonable. It can be deemed unreasonable if the supply of government institutions outweighs the external effective demand.

*q* indicates the input amount of administrative resources; *R* represents administrative output; *C* represents EMC; *Z* represents administrative efficiency; *R*=*f*_*i*_(*q*) function represents the functional relationship between administrative output and input of administrative resources. The function *C*=*g*_*i*_(*q*) represents EMC's functional relationship about the input of administrative resources. Establish the following mathematical model formula:

(1) $$\begin{array}{c} Z_{i}=\frac{f_{\left(t_{i}\right)}\left(q\right)}{g_{\left(t_{i}\right)}\left(q\right)},\;i=1,2,\ldots ,N,\;Q_{t_{i-1}}\leq Q\leq Q_{t_{i}}. \end{array}$$

Dynamic cost management implementation helps modernize the cost management concept. Saving becomes the primary strategy for cost reduction in traditional cost management because it is the goal of the practice. Giving customers more use value for the same price or the same use value for less money is how a company gains a competitive edge in the market. The overall business strategy and competitive strategy of an organization determine the cost strategy it adopts, and cost management should support overall enterprise management.

Administrative costs (including funds provided by state organs and subsidies for the operations of nongovernmental organizations) and diplomatic costs are included in the budget expenses needed for the operations of state organs of power and administrative organs. EMC includes a significant portion of administrative costs, which is a reflection of China's problem with an overabundance of administrative institutions on all levels. In accordance with the norms of the current democratic system, officials maximize the departmental budget and always work to further their own interests. The market mechanism, which predicts that it will take some time for our government to reach a reasonable and moderate scale, cannot be fully credited. It will be crucial to keep EMC functioning at a high level because it is a long-lasting phenomenon.

In this work, the graph of mathematical model adopts object-oriented design method. The main idea is to establish a mathematical model by taking the real physical object as an independent module, and all other activities are carried out around this module, which is implied in the graphic network. The overall structure of the system is shown in Figure 1.

The graphic editing subsystem draws the corresponding flow model diagram according to the user's drag and drop, and informs the algorithm configuration system to generate the corresponding mathematical model. When the user modifies the model graph, the graph editing subsystem transmits the graph changes with time to the algorithm configuration system, which modifies and adjusts the model accordingly and presents the modified results to the user.

*A* is the *n* × *n* matrix composed of *a*_*ij*_, which represents the corresponding relationship matrix between self-produced products, including consumption relationship. *B* is a *m* × *n*-order matrix composed of *b*_*kj*_, which represents the fixed consumption relationship required to produce a certain unit product.

Available:

(2) $$\begin{array}{c} {\left(I-A\right)}^{-1}Y=RY=X. \end{array}$$

Substitute it into equation (1) to get

(3) $$\begin{array}{c} B{\left(I-A\right)}^{-1}Y=QY=Z. \end{array}$$

The complete consumption coefficient table is formed by *R*=(*I* − *A*)^−1^,  *Q*=*B∗*(*I* − *A*)^−1^ matrix. The *R* matrix and *Q* matrix can be used to calculate the dynamic cost of a specific single product.

### 3.2. Implementation of Cost Quick Control Based on BSC

Compared with the traditional performance evaluation system, BSC puts more emphasis on the factors that create long-term economic benefits, such as customers, internal processes, and learning and growth of enterprises. The main features of BSC are as follows:

1. Focus on customers. Meet and retain existing customers in the target market classification, and strive for new customers.
2. Pay attention to the learning and growth of the organization. BSC emphasizes that through organizational learning, skilled and willing employees can be trained, and strategic information contact channels can be provided to make the organization grow continuously.
3. BSC pays attention to the value-creating activities of highly skilled and motivated enterprise personnel. On the one hand, it keeps paying attention to short-term performance from a financial perspective, on the other hand, it can clearly reveal how to ensure long-term financial and competitive performance.

BSC-based control system subdivides cost management objectives around the four key dimensions of BSC, comprehensively analyzes the specific relationship between management objectives and functions, and makes qualitative analysis, quantitative analysis, and model construction to analyze the role of the system. Therefore, it is necessary to establish a scientific and reasonable public budget system, optimize and adjust the public budget structure, gradually increase the financial investment in public services related to people's livelihood, such as education, health, and social security, and reduce the administrative operation cost. Government agencies, that make them more suitable for the needs of the transformation of government functions, and invest limited funds in places where they are most needed.

Whether it is a small government + a big society, or a big company + a small company, such incompatibility will also produce high social costs. High cost means less profit, more input, and less output. Because of the serious imbalance between the non-production management system and the production management system, the government cannot support the development of the big society, the supply and demand of government public goods are out of balance, and the scale of the government does not adapt to the social and economic development. The government pursues the general trend of budget maximization, ignoring the right of ordinary people to know and benefit from the public financial system, and is unable to obtain effective social supervision. In practice, due to the objective reality of the inherent defects of China's government budget management system, rent-seeking budgets will always appear in government departments, which will inevitably lead to the expansion and waste of EMC, thus leading to high costs.

BSC-based EMC control can find ways to reduce costs and improve profitability in the specific implementation process, thus promoting the effective combination of cost management and government strategy, and further solving the problem that traditional cost management does not attach importance to government strategy. Establish an EMC control system under BSC, as shown in Figure 2.

To control the cost from the strategic level and apply BSC to cost management, the key factor is to follow the four dimensions of BSC. Based on different perspectives of four dimensions in BSC, the corresponding EMC control objectives are decomposed into corresponding cost indicators, and scientific application analysis can improve the efficiency of EMC control.

The cost optimization control method is to redetermine the minimum controllable target cost through cost optimization on the premise of determining the initial target cost. For this problem, as the number of processes increases, the search space is also greatly expanded. It is difficult or even impossible to find its optimal solution on today's computer, and GA is one of the best tools to find this satisfactory solution. In engineering practice, the target quality level is usually given to find the optimal cost of the system. Combined with the above quality cost relationship model, the objective function of quality cost optimization based on GA is

(4) $$\begin{array}{c} y=\min\sum_{i=1}^{n}\left\{C_{b}\left(i\right)\left[\omega_{1}{\left(tg\left(\left(\frac{\pi }{2}\right)*R\left(i\right)\right)\right)}^{K_{1}}+\omega_{2}{\left(ctg\left(\left(\frac{\pi }{2}\right)*R\left(i\right)\right)\right)}^{K_{2}}\right]\right\}. \end{array}$$

Among them, *C*(*i*) is the total cost of quality. The first item in the formula is the pre-evaluation cost, and the second item is the failure cost; *C*_*b*_(*i*) is the basic cost value of the *i*th subsystem; *ω*_1_, *ω*_2_ is the ratio of pre-appraisal cost and loss cost to total quality cost; *R*(*i*) is the reliability of the *i*th subsystem; and *K*_*i*_(*i* − 1,2) is the cost growth index.

Two different individuals, which are all composed of the normal duration method and the limit time method, are generated, respectively, and their respective normal and limit total construction periods are obtained. The shortest distance *d*_*i*_ between each individual and the lower envelope is calculated, which represents the smallest distance of each line segment. It can be obtained by the following formula:

(5) $$\begin{array}{c} f_{i}=d_{\max}-d_{i},\\ p_{i}=\frac{f_{i}}{\sum f_{i}}. \end{array}$$

Among them, *d*_max_=max(*d*_*i*_),  *i*=1,2,…, *N*.

The elements stored in the cross-database designed in this article are selected by tournament selection method. By changing the scale of the league, we can ensure that the individuals who enter the cross-database are in line with the evolutionary characteristics. When creating the cross-library, the league size of the tournament selection method is

(6) $$\begin{array}{c} r\left(t\right)=\beta_{2}\times N\frac{\alpha \left(t\right)}{\alpha_{\max}}, \end{array}$$

*r*(*t*) is an integer rounded down, which indicates the league scale of the tournament selection method when the *t*-generation cross-database is created, and the minimum value of *r*(*t*) is defined as *N*/20; *β*_2_ is the adjustment coefficient, taking the value [0.05, 0.2].

The core idea of parallel mutation is to perform several completely different mutation operations at the same time, and then select the most appropriate operation result from all the obtained mutation results as the final mutation result of the algorithm. Assuming that the result of a mutation in the *t* − 1-generation population is *x*_*i*_^*t*^, the specific rules of parallel mutation are as follows:

(7) $$\begin{array}{c} x_{i}^{t}=k\times \left(x_{\max}-x_{\min}\right)+x_{\min}. \end{array}$$

Because this mutation method has certain effect in jumping out of the local optimal solution and maintaining the diversity of the population, it is an important condition to ensure the global convergence of the algorithm, so it is retained as a mutation rule in parallel mutation.

(8) $$\begin{array}{c} x_{2}^{t}=k\times \left(x_{\max}^{t-1}-x_{\text{best}}^{t-1}\right)+x_{\text{best}}^{t-1}. \end{array}$$

Among them, *x*_2_^*t*^ is the result of mutation according to the second method, and *x*_best_^*t*−1^ is the individual with the best individual fitness value in the *t* − 1-generation population before the mutation operation; *x*_max_^*t*−1^ is the individual with the largest actual value in the *t* − 1 generation group.

Synthesizing all the improvements of genetic operation proposed in this chapter, this article proposes a GA based on cross-database and parallel mutation, and its specific algorithm flow is shown in Figure 3.

The algorithm steps are as follows:

1. Setting parameters and initializing the population.
2. Decoding chromosomes and selecting regenerated individuals according to fitness.
3. Determining the variation mode and performing variation according to the variation probability.
4. The evolution algebra is added with 1, and the new generation population generated by cross mutation returns to step (2).
5. Record the current evolutionary population and evaluate the current optimal individual.
6. The path population obtained by searching is saved, and the algorithm ends to compare all feasible solutions and output the optimal solution.

## 4. Experiment and Results

According to our previous BSC-based government EMC rapid control index system, this AHP (analytic hierarchy process) model has been basically formed, and the hierarchical model is divided into three levels. In this study, the AHP software is used to establish a fast government cost control model. Through the statistics of 15 expert consultation questionnaires, the expert judgment matrix is normalized by normalization method. The analysis of the judgment results of each expert on the first-level indicators is shown in Figure 4, and the consistency test results are shown in Figure 5.

As can be seen from Figure 4, the CI of the consistency test results of 15 experts' judgments on the first-class indicators are all less than 0.1, and similarly, the CR is all less than 0.1, all of which meet the test requirements. There are two main types of institutional change, according to new institutional economics: induced institutional change and compulsory institutional change. When we look at how China's government system is changing, we can say that two paths are being taken simultaneously, but the second one is the main one. Our institutional change must be fueled by the power and might of the state because the cause is the executive branch's own strength and inertia. Social media organizations primarily regulate the self-discipline and management practices of governments in areas like technical standards for generic products, employee certification of qualifications and professional title evaluation, industry statistics, and basic information research, among others. The community is primarily responsible for the self-regulating function of the masses, and the masses independently handle issues that fall under their purview of mass autonomy.

This shows that the judgment matrix meets the consistency requirement and is acceptable, and the obtained weight is valid, which shows that the judgment matrix selected before is reasonable, so we can proceed to the next step. The weights of the second-level indicators are shown in Table 1 and Figure 6.

From the financial point of view, the rate of return on investment and the growth rate of output value accounts for a very large proportion, which shows that from the traditional financial point of view, enterprises should attach importance to their investment and output value. On the other hand, the more enterprises attach importance to it, the more they usually invest, and the greater the space for cost control. If a certain cost can attract new customers or retain old customers, then these costs are all worthwhile. Therefore, cost and control are not absolute, and it is necessary to distinguish the relationship between investment and return.

By looking at the representative indicators from the four BSC areas, we can intuitively determine which indicators carry the most weight and which areas businesses should focus on in their daily operations. Find out the customer company's weaknesses, build and produce in accordance with the needs of the customer, and realize the reasonable colocation of investment and acquisition, for instance, be mindful of any potential space during internal processes such as design, procurement, and production. In order to better control and manage costs, we must focus on the specifics of consumption costs during this process. In internal management, there are some closed issues. It is challenging to address some issues comprehensively, even when all departments can communicate to an extent. People tend to believe that planning manages overall planning and management while finance manages financial indicators. As a result, there will be issues like a lengthy reporting period and poor efficiency. The implementation of process control analysis and evaluation will simultaneously depend on numerous human factors.

Input the conditions of the project into the compiled program file, and take *M* = 150, *T* = 200, *ω*_1_ = *ω*_2_, *λ*_1_ = 0.2, and *λ*_2_ = 0.6. After running the target cost optimization configuration program based on GA, the optimized configuration results are shown in Figure 7.

It can be seen that the result of the optimized configuration scheme provided is relatively intuitive. Through the analysis of the above two schemes, the first scheme is inferior to the second scheme in terms of construction period and total project cost, so the second scheme can be taken as the final control scheme. According to the technical level and management level of the project department, the configuration of construction machinery, the intensity of market changes, and other factors, different choices should be made. These are all factors that affect the formula and must be fully considered when determining the specific control scheme.

To verify the general performance of the method proposed in this article, the commonly used Shubert test function is selected, and each test function is set with a threshold value. When the threshold value is reached in the specified algebra, the algorithm is considered to be convergent. Algorithms proposed in refs 15, 17, 19 and the algorithm proposed in this article are used to simulate and compare test functions (the overall size of each example is 200, and the test is repeated 100 times). The performance statistics results of different algorithms of Shubert function are shown in Table 2, and the performance comparison results of different algorithms are shown in Figure 8.

In terms of average convergence algebra and convergence time, the performances of algorithms in ref [17] and ref [19] are obviously better than those of ref [15], and their results are similar. However, the algorithm proposed in this article has the best performance, with the least convergence algebra and the most convergence times, because the cross-parallel basis mutation can update the population to the direction of optimal solution, and always keep good optimization ability.

The algorithm in this article has the shortest average convergence time (0.186 s), ranking it as the least. The variances obtained by the five algorithms have the same order of magnitude in terms of population fitness, but this algorithm's variance is the smallest and its variance of population fitness is 288.19, indicating that the overuse of algorithms in this study may result in a decline in population diversity due to an excess of superior individuals in the cross-database elements. Establishing an effective reward and punishment system as well as carrying out a reasonable and scientific cost control inspection and evaluation on the government are required in order to guarantee the long-term stable operation and development of the government's EMC control system. Each department should rank the projects in order of importance when creating the departmental budget. The government can make decisions based on the relative importance of the projects from different departments, allocate scarce resources to projects that are urgently needed, focus on important work, and increase efficiency. In terms of the use of funds, improving the financial control function can both standardize the internal management of the financial department and oversee the expense department's budget execution function. Financial engineering also effectively encourages the openness of government affairs and the development of government transparency by giving the public a way to participate directly in the management and oversight of the government's finances.

## 5. Conclusions

EMC's management and control is not simply to reduce the total cost, but to deeply analyze the composition of the cost, analyze the reasons and trends of its growth, and make it meet the requirements of government functions and the needs of economic and social development. Through BSC-based EMC governance, the original fast control mode is broken, not only from the financial point of view but also from the customer's point of view, internal process point of view, learning and growth point of view. This article puts forward the method of BSC to solve the government EMC problem. The central idea of BSC is to focus on the government's development strategy, promote each other and balance each other through the construction of financial, customer, internal process, learning, and growth indicators. GA is applied to solve the problem of optimal allocation of construction project's time limit for each process, quality level of corresponding process, and cost value. Through continuous analysis, the target value is adjusted so that the process cost and the total project cost are always under optimal control. Simulation results show that the algorithm proposed in this article can overcome the problems of slow convergence speed and low convergence accuracy of GA, and it can perform well in practical applications.

## Figures and Tables

**Figure 1:** Graphical design structure.

**Figure 2:** The architecture of EMC control based on BSC.

**Figure 3:** Algorithm flow.

**Figure 4:** Judgment of each expert in the first-level index.

**Figure 5:** Consistency test result.

**Figure 6:** The second layer index weight radar chart.

**Figure 7:** Optimization result.

**Figure 8:** Performance comparison of different algorithms.

**Table 1:** BSC index system.

The second-level index	Level 2 index weight (%)
Rate of return on investment	15.36
Income growth rate	7.01
Output value growth rate	4.31
Customer satisfaction	13.28
Customer value change rate	14.57
Employee training rate	5.52
Product innovation rate	1.33

**Table 2:** Statistical results of different algorithm performances.

Algorithm	Average convergence algebra	Convergence times	Average solution	Average convergence time of algorithm/s	Variance of final population fitness
Ref [15]	51.23	40	−188.24	0.236	472.15
Ref [17]	44.07	46	−188.24	0.214	478.96
Ref [19]	36.98	46	−188.01	0.208	613.28
Algorithm in this article	22.01	48	−88.63	0.186	288.19

## Data Availability

The data used to support the findings of this study are available from the corresponding author upon request.
